RETRACTED

# The Optos 200Tx Scanning Laser Ophthalmoscope Application in Retinoblastoma Patients' Follow-Up

**DOI:** 10.1155/2022/5422360

**Published:** 2022-08-11

**Authors:** Xuehao Cui, Xunda Ji, Yan Shao, Peiquan Zhao, Xiaorong Li

**Affiliations:** ^1^Tianjin Key Laboratory of Retinal Functions and Diseases, Tianjin International Joint Research and Development Centre of Ophthalmology and Vision Science, Eye Institute and School of Optometry, Tianjin Medical University Eye Hospital, 300384, China; ^2^Xinhua Hospital Affiliated to Shanghai Jiaotong University School of Medicine 200092, Department of Ophthalmology, China

## Abstract

**Methods:**

A total of 1134 examinations with Optomap 200Tx were performed for 318 children who were clinically diagnosed with RB in the Ophthalmology Department of Tianjin Medical University Eye Hospital, China, between July 2015 and July 2017, and achieved stable disease lasting for more than 6 months after combined treatment. The children received examinations every 1-12 months (mean 4 months), initially at 31 months to 15 years of age (mean 51 months), and were given a full eye examination under anesthesia (EUA) immediately if recurrent tumor, recurrent vitreous seeding (VS), or recurrent subretinal seeding (SRS) was detected, or in the next follow-up visit if no abnormality was detected, and early treatment was performed when the lesion was confirmed.

**Results:**

Recurrence was detected in 4 children in the examination with Optomap 200Tx, including 2 cases of recurrent vitreous seeding (VS) and 2 cases of recurrent subretinal seeding (SRS), which were confirmed by EUA and well controlled after early treatment.

**Conclusion:**

The use of Optomap 200Tx in the long-term following up of patients with RB reduces the number of eye examinations under general anesthesia (EUA), increases the time between EUAs, and protects children from exposure to the adverse effects of general anesthetics. Optomap 200Tx can detect recurrent tumor and recurrent seeding, allowing for early treatment which produces better outcomes.

## 1. Introduction

Retinoblastoma (RB) is the most common primary malignant tumor seen in infants and children, with an incidence rate of one in 15-20000 children [1–5]. The strategy of using combined systemic chemotherapy, intra-arterial chemotherapy (IAC), and topical therapy has achieved a 5-year survival rate of 95% and partial vision reservation in pediatric patients with intraocular RB in recent years [6, 7]. Regular follow-up in the course of treatment is important for early detection of recurrent tumors and seeding. It also facilitates to understand the disease progression and evaluate the effects of treatment, providing clinical basis for further treatment [7].

RETRACTED

Examination under general anesthesia (EUA) is the conventional method for follow-up of RB patients [8]. As most of the RB patients are infants or children, general anesthesia may put the children at greater risk and affect their growth and development [8]. Backeljauw et al. [9] reported a control study involving 53 children who had received general anesthesia before 4 years of age and 53 who did not. Children in the experimental group scored lower in language development and listening comprehension ability than the control group and showed lower grey matter density in head magnetic resonance imaging (MRI) [9]. The United States' Food and Drug Administration (FDA) issued a warning in December 2016 that repeated or long-time use of general anesthetics or sedative in women in the third trimester or in children under 3 years of age may compromise the brain development of the fetuses and children [10]. Recent studies on animals showed that exposure of developing brains to anesthetics may cause extensive neuron apoptosis and neurodegeneration leading to neuropsychological or behavioral developmental disorders [11].

Optomap 200Tx is an emerging fundoscopy system, which has such advantages as a broader view, no needs for anesthesia, and increased convenience as compared to EUA. This study was aimed at observing and evaluating the application value of Optos 200Tx scanning laser ophthalmoscope (Optomap 200Tx) in the long-term follow-up of patients with RB who achieves stable disease after treatment.

## 2. Materials and Methods

### 2.1. Study Subjects

This retrospective study was performed on the data of 318 children who were clinically diagnosed with RB in the Ophthalmology Department of Tianjin Medical University Eye Hospital, China, between July 2015 and July 2017. Those patients who achieved stable disease lasting for more than 6 months after combined treatment and received examinations with Optomap 200Tx during their follow-ups were included in the study. Data of those patients who had incomplete information or missed the follow-up were excluded from the study. This study was approved by the ethics committee of the Tianjin Medical University Eye Hospital, China.

### 2.2. Examination with Optomap 200Tx

Prior to the examination with Optomap 200Tx, 5 images of the fundus (posterior pole, nasal, superior, inferior, and temporal side) were taken by a medical professional after the use of mydriatics in darkroom. The images were then sent to the information system of the hospital for reading and interpretation by doctors with specialization in RB, and the children's families were informed of the results. The RB staging was assigned according to the International Retinoblastoma Staging System as stage A–stage E.

RETRACTED

### 2.3. Statistical Analysis

SPSS software (version 23.0) was used for data analysis in the study. The measurement data were expressed as Mean ± SD. Count data were expressed as numbers or percentages.

## 3. Results

The data of 318 patients including 168 males and 150 females were analyzed. One hundred and two (102) children had unilateral and 216 children had bilateral tumors. According to the International Retinoblastoma Staging System, 35 cases were in stage A, 53 in stage B, 102 in stage C, 84 in stage D, and 44 in stage E. The children received a total of 1-8 (mean 3.57) examinations every 1-12 months (mean 4 months). A total of 1134 examinations with Optomap 200Tx were performed for 318 children with RB.

During the examination with Optomap 200Tx, presence of recurrent tumor and seeding, which requires early treatment (Figures 1(a) and 1(b)); activity of vitreous or subretinal seeding (Figure 1(c)); extent of calcification of tumors and stability of fish-like tumors (Figure 1(d)); presence of new tumors in the contralateral eye of children with unilateral RB (Figures 1(e) and 1(f)); and presence of complications such as retinal detachment, fundus angiopathy, and choroidal atrophy (Figure 1(g)), was observed. The children were given EUA immediately if recurrence was detected in the examination with Optomap 200Tx, or in the next follow-up visit if no recurrence was detected, in order to confirm the lesion.

Recurrence was detected in 4 children, which were confirmed by EUA and well controlled after early treatment. Examination with Optomap 200Tx demonstrated inactive VS and SRS, stable fish-like tumor, which were confirmed by EUA in the next follow-up visit. New oncogenesis was not found in the examination of the contralateral eye of children with unilateral RB with Optomap 200Tx. Retinal detachment was observed in 1 child and was successfully restored after surgical treatment. According to Table 1, the sensitivity and specificity of Optomap 200Tx to recurrent VS and SRS was 100% and 100%, respectively. However, statistical analysis showed that there were few cases of recurrence. The reason for the low incidence of recurrence in follow-ups could be due to the fact that examination with Optomap 200Tx was performed for children who achieved stable disease lasting for more than 6 months (6-28 months, mean 14 months) after combined treatment.

## 4. Discussion

In recent years, Optomap 200Tx is widely used in the fundoscopy of patients with various retinal diseases, including diabetic retinopathy [12], age-related macular degeneration [13], retinal pigment degeneration [14], and retinopathy in children [15], and is considered an effective means of examination. Compared with EUA, Optomap 200Tx is considered superior due to several reasons including its ultrawide field of view (200°) which is capable of photographing areas from the posterior pole to the peripheral areas. In addition, it allows clear display of tumors around the retina, such as recurrent tumor and seeding in the follow-up examination of RB patients. Moreover, there is no need of anesthesia, which avoids the risks caused by anesthesia and reduces the times of general anesthesia in the long-term follow-up and the adverse effect of general anesthesia on the growth and development of children. It is easier to operate than EUA and more suitable for long-term follow-up of patients. It has a wider angle in autofluorescence and fundus fluorescein angiography than conventional machines [8]. It takes only 0.3 s to complete the photographing, which reduces the difficulties due to poor cooperation of young child with RB. It does not contact with the eyeball, which avoided infection, corneal injury, subconjunctival hemorrhage, and other complications of the eyes. It provides high-resolution images, which increases the accuracy of the physician's judgement, and allows use in remote consultation and academic exchange. It is inexpensive and saves the expenses for anesthesia and related examinations, as well as the fasting before and after anesthesia. The examination is normally completed within 10 minutes.

RETRACTED

Still, Optomap 200Tx has some limitations and shortcomings including extremely peripheral areas are difficult to photograph, for example, recurrence near the ora serrata cannot be seen. In addition, it is not effective in detecting some retinopathies. Mackenzie [16] found that Optomap 200Tx has a low sensitivity to disorders in pre-equatorial retina. It requires active cooperation of the children, and thus is not suitable for children under 3 years of age or uncooperative children. The quality of image will be poor when the children are not cooperative. In EUA, the operator may press the eyeball to view the extremely peripheral retina, and steadier photographing is obtained as the children are in general anesthesia, which is not possible in examination with Optomap 200Tx. Therefore, Optomap 200Tx cannot completely replace fundus under general anesthesia. Our strategy is to use Optomap 200Tx and EUA alternately. This study suggests that Optomap 200Tx can be used in the long-term following up of patients with RB who achieve stable disease, to effectively monitor changes in the fundus, detect recurrent tumors and fundus complications, increase the time between fundus examinations under general anesthesia, and reduce the adverse effect of anesthesia on the growth and development of THE children. However, Optomap 200Tx cannot completely replace EUA, but can be used as a supplementary of EUA in the long-term follow-up of children with RB.

RETRACTED

## 5. Conclusion

Most of the RB patients are infants or children, and general anesthesia for examination often put the children at great risk and affect their growth and development. This retrospective study was aimed at observing and evaluating the application value of Optos 200Tx scanning laser ophthalmoscope (Optomap 200Tx) in the long-term follow-up of patients with RB who achieves stable disease after treatment. A total of 1134 examinations with Optomap 200Tx were performed for 318 children who were clinically diagnosed with RB and achieved stable disease lasting for more than 6 months after combined treatment. Recurrence was detected in 4 children in the examination with Optomap 200Tx, including 2 cases of recurrent vitreous seeding (VS) and 2 cases of recurrent subretinal seeding (SRS), which were confirmed by EUA and well controlled after early treatment. The use of Optomap 200Tx in the long-term following up of patients with RB reduces the number of eye examinations under general anesthesia (EUA), increases the time between EUAs, and protects children from exposure to the adverse effects of general anesthetics. Optomap 200Tx can detect recurrent tumor and recurrent seeding, allowing for early treatment which produces better outcomes.

## Figures and Tables

**Figure 1:** Examples of main observations in the examination with Optomap 200Tx. (a) Recurrent tumor above the macula lutea. (b) Significantly shrank recurrent tumor after a intra-arterial chemotherapy. (c) Large amount of inactive VS. (d) Partial calcification of the tumor beside the optic papilla, with neovascularization on the surface, which obscures the macular area. (e) Affected eye of child with unilateral RB. (f) Contralateral eye of child with unilateral RB without any abnormality. (g) Retinal detachment seen in the temporal side.

**Table 1:** Sensitivity and specificity of Optomap 200Tx to recurrent VS and SRS.

Examination methods	Optomap 200TX	EUA
VS	2	2
SRS	2	2
Recurrent tumor	0	0
Stable	1130	1130
Total	1134	1134

## Data Availability

Data will be provided upon reasonable request to the corresponding author.
